# Prognostic Analysis of Liver Cirrhosis Patients with Cerebral Infarction and/or Gastrointestinal Hemorrhage: A Retrospective Cohort Study

**DOI:** 10.1155/2022/2566746

**Published:** 2022-08-04

**Authors:** Dianqiang Lu, Zhengyan Jiang, Xuezhen Zhai, Zhiguang Sun

**Affiliations:** ^1^Center of Digestive Endoscopy, The Second Affiliated Hospital of Nanjing University of Chinese Medicine, Nanjing 210017, China; ^2^Huaiyin Hospital of Huai'an City, Huaian 223300, China; ^3^Nanjing University of Chinese Medicine, Nanjing 210017, China

## Abstract

**Background:**

To explore the risk factors of gastrointestinal hemorrhage and/or cerebral infarction complications in liver cirrhosis and provide evidence for early prevention, clinical diagnosis, and treatment of liver cirrhosis.

**Methods:**

200 liver cirrhosis patients were analyzed: liver cirrhosis (*n* = 78), liver cirrhosis complicated with cerebral infarction (*n* = 43), liver cirrhosis complicated with gastrointestinal hemorrhage (*n* = 57), and liver cirrhosis complicated with gastrointestinal hemorrhage and cerebral infarction (*n* = 22). The incidence of disease in each group of patients at different times was calculated. Multivariate logistic regression was used to analyze the risk factors of liver cirrhosis patients with gastrointestinal hemorrhage and cerebral infarction. After 12 months of follow-up, the mortality rate of each group was calculated.

**Results:**

The incidences of gastrointestinal hemorrhage, cerebral infarction, and gastrointestinal hemorrhage combined with cerebral infarction in patients with liver cirrhosis were 21.5%, 28.5%, and 11%, respectively. The width of the portal vein, D-2 polymer, albumin (ALB), and hemoglobin (Hb) were predictors of gastrointestinal hemorrhage and cerebral infarction in patients with liver cirrhosis. Age, hypertension, bleeding history, infection, portal vein width, and D-2 polymer were confirmed as risk factors for gastrointestinal hemorrhage and cerebral infarction in patients with liver cirrhosis. ALB and Hb were independent protective factors. Patients with liver cirrhosis and gastrointestinal hemorrhage with cerebral infarction had the worst survival.

**Conclusion:**

Age, hypertension, bleeding history, infection, portal vein width, and D-2 polymer are all independent risk factors for gastrointestinal bleeding and cerebral infarction, while ALB and Hb are independent protective factors.

## 1. Introduction

Liver cirrhosis is one of the most common chronic liver diseases. It is caused by long-term repeated actions of various etiologies on the liver resulting in large-scale degeneration and necrosis of the liver cells. The diffuse proliferation of the liver fibrous tissue forms pseudolobules, which destroy the liver cell structure eventually leading to severe liver function decompensation in the late stage [1, 2]. Epidemiological studies have shown that recently, the incidence and mortality of liver cirrhosis have been increasing annually, with more than 1 million deaths each year, making it the 14th leading cause of death worldwide [3]. The causes of liver cirrhosis mainly include alcoholism, hepatitis C virus (HCV), nonalcoholic fatty liver disease, and posthepatitis cirrhosis [4, 5]. Liver cirrhosis can be subdivided into different clinical prognostic stages with 1-year mortality varying from 1% to 27% depending on the stage [6]. Due to the lack of specific symptoms of compensated liver cirrhosis, at the time of diagnosis, most patients are already in the decompensated stage and have liver damage and portal hypertension-related complications, such as gastrointestinal hemorrhage, ascites, pleural effusion, secondary infection, portal vein thrombosis, hepatic encephalopathy, hepatorenal syndrome, hepatopulmonary syndrome, and primary liver cancer [2, 7], leading to poor prognosis. In particular, patients with liver cirrhosis are prone to extrahepatic hemorrhagic and thrombotic complications [8].

Upper gastrointestinal hemorrhage is one of the most common extrahepatic hemorrhagic complications and is associated with high mortality in patients with liver cirrhosis [9]. It is reported that approximately 30% of patients with liver cirrhosis will have an upper gastrointestinal hemorrhage in the late stage of the disease. The level of hemorrhage ranges from mild, presenting with melena, to severe gastrointestinal hemorrhage which leads to a life-threatening sharp drop in circulating blood volume [9, 10].

Cerebral infarction, a thrombotic complication, is the second leading cause of death globally [11, 12]. According to the 2019 China Health Statistics Summary data, in 2018, more than 20% of Chinese residents died of cerebrovascular disease, which means that stroke accounted for at least 1 out of every 5 deaths [12]. Patients with liver cirrhosis are prone to coagulation complications [13]. In particular, at the decompensated liver cirrhosis stage, patients often experience bleeding in different sites at different degrees of severity, prolonged conventional prothrombin time (PT), and activated partial prothrombin time (APTT). Consequently, in the past, even scholars believed that liver cirrhosis is a state of “automatic anticoagulation” and is not prone to thrombosis [14]. However, studies suggest that thrombotic events in patients with liver cirrhosis are not uncommon [15, 16] and a recent study has shown that liver cirrhosis is hypercoagulable and prone to thrombosis [16].

Despite the associated high risk of mortality and the significant incidence in patients with liver cirrhosis, there are a few studies on liver cirrhosis gastrointestinal hemorrhage and/or cerebral infarction complications. Therefore, this study will explore the prognosis of patients with liver cirrhosis combined with gastrointestinal hemorrhage and/or cerebral infarction and provide a theoretical basis for clinical decision-making.

## 2. Method

### 2.1. Research Subjects

A total of 200 hospitalized liver cirrhosis patients who received treatment in our hospital from May 2016 to August 2019 were retrospectively analyzed.

#### 2.1.1. Inclusion Criteria

Inclusion criteria are as follows: (1) patients with liver function decline (presenting with fatigue, anorexia, etc.) and portal hypertension (presenting with splenomegaly, ascites, etc.) and related clinical manifestations; (2) reduced serum albumin content (ALB < 30 g/L), elevated serum total bilirubin (TBIL > 17.1 mmol/L); (3) abdominal CT, MRI, and B-ultrasound suggest hepatomegaly or liver shrinkage, hepatic portal enlargement, hepatic lobe disproportional, splenomegaly, and portal vein, hepatic vein, or collateral vessels widening and other imaging manifestations, clinically confirmed patients with liver cirrhosis; (4) after diagnosis, some patients were accompanied by gastrointestinal hemorrhage and/or cerebral infarction; (5) patients who gave informed consent and volunteered to participate in this study.

#### 2.1.2. Exclusion Criteria

Exclusion criteria are as follows: (1) patients with malignant tumors; (2) patients with mental illnesses; (3) patients with severe liver and kidney dysfunction; (4) patients with other severe cardiovascular and cerebrovascular diseases.

According to clinical complications, patients were divided into 4 groups: liver cirrhosis group (*n* = 78), liver cirrhosis complicated with cerebral infarction group (*n* = 43), liver cirrhosis complicated with gastrointestinal hemorrhage group (*n* = 57), and liver cirrhosis complicated with gastrointestinal hemorrhage and cerebral infarction group (*n* = 22). The Second Affiliated Hospital of Nanjing University of Chinese Medicine (No. SEZLC20211201) Ethics Committee approved this study.

### 2.2. Patient General Data Collection

Clinical baseline characteristics of all the patients including age, gender, height, weight, duration of liver cirrhosis, heart rate before admission, blood pressure, past medical history, smoking, alcohol consumption, and the presence or absence of primary/complications were collected.

### 2.3. Analysis of the Characteristics of Patients' Clinical Indicators

The clinical parameters of liver cirrhosis patients with gastrointestinal hemorrhage and cerebral infarction were recorded and compared. Their parameters were portal vein width, PT, D-dimer, fibrinogen, triglycerides (TG), total cholesterol (TC), low-density lipoprotein (LDL-C), alanine aminotransferase (ALT), aspartate aminotransferase (AST), ALB, TBIL, direct bilirubin (DBIL), blood urea nitrogen (BUN), creatinine (Cr), C-reactive protein (CRP), white blood cell count (WBC), platelet count (PLT), and hemoglobin (Hb).

### 2.4. Complication Rate

The patients were followed up at 3, 6, 9, and 12 months after treatment, and the incidence rate of gastrointestinal hemorrhage, cerebral infarction, and gastrointestinal hemorrhage with cerebral infarction in patients with liver cirrhosis for each period was calculated.

### 2.5. Statistical Analysis

The experimental data were analyzed using SPSS 22.0 software. The measurement data were expressed by mean ± standard deviation (mean ± SD); the comparison between two groups was done by the *t*-test, and the comparison between multiple groups was done by single-factor analysis; enumeration data were expressed by *n* (%), and the comparison between groups was done by the chi-square test. Single-factor and multivariate logistic regression was used to analyze the influencing factors of liver cirrhosis with gastrointestinal hemorrhage and cerebral infarction; Kaplan-Meier was used to draw the survival curves, and the survival rate between groups was compared by log-rank test. *P* < 0.05 was considered to indicate a statistically significant difference.

## 3. Result

### 3.1. General Patients' Information

A total of 200 patients were enrolled. A comparison of the general data between the four groups only showed significant differences in age, alcohol consumption, bleeding history, and infection rate (*P* < 0.05). There were no statistically significant differences in other indicators (such as gender, height, and weight) between the groups (Table 1). These results suggest that age, alcohol consumption, bleeding history, and infection rates may be related to the occurrence of complications in patients with liver cirrhosis. A flowchart of this research study design is presented in Figure 1.

### 3.2. Comparison of Patients' Clinical Characteristics

The clinical characteristics of the four groups of patients were compared. The results showed significant differences in the portal vein width, D-2 polymer, ALB, and Hb among the four groups. The width of the portal vein of the patients in the cerebral infarction, gastrointestinal hemorrhage, and gastrointestinal hemorrhage with cerebral infarction groups was significantly higher than that of the liver cirrhosis group, while the D-2 polymers of patients in the cerebral infarction and gastrointestinal hemorrhage with cerebral infarction groups were significantly higher those in the liver cirrhosis and gastrointestinal groups. The ALB and Hb of the three complication groups were also significantly lower than those of the cirrhosis group (Table 2).

### 3.3. Comparison of Patients' Mortality Rate

The mortality of each group of patients after 12 months of follow-up was analyzed. The results showed that the gastrointestinal hemorrhage with cerebral infarction group had the worst survival rates (13/22, the mortality rate was 59.1%), while the liver cirrhosis group had the best survival rate (0/41, 0% mortality rate) (Figure 2). These results show that patients with liver cirrhosis and gastrointestinal hemorrhage with cerebral infarction have the worst prognosis.

### 3.4. The Incidence of Complications in the Three Complication Groups of Patients with Liver Cirrhosis

Patients with liver cirrhosis were followed up at 3, 6, 9, and 12 months after surgery, and the incidence of complications in patients with liver cirrhosis at different time periods was recorded. The results showed that the incidence of gastrointestinal hemorrhage was the highest in the 3, 6, 9, and 12 months of follow-up. After 12 months, 43 patients had cerebral infarction, 57 had gastrointestinal hemorrhaging, and 22 had gastrointestinal hemorrhage with cerebral infarction (Figure 3).

### 3.5. Single-Factor Logistic Analysis of Influencing Factors in Patients with Liver Cirrhosis with Gastrointestinal Hemorrhage and Cerebral Infarction

Single-factor logistic analysis was used to analyze the influencing factors of gastrointestinal hemorrhage and cerebral infarction in patients with liver cirrhosis. First, the baseline characteristics of patients in the liver cirrhosis group and those in the gastrointestinal hemorrhage with cerebral infarction group were analyzed. The results showed significant differences in age, hypertension, alcohol consumption, bleeding history, and infection between the two groups (*P* < 0.05, Table 3). This suggested that these may be influencing factors of gastrointestinal hemorrhage and cerebral infarction in patients with liver cirrhosis. Further, a single-factor analysis of the clinical indicators between the two groups showed statistically significant differences in the portal vein width, D-2 polymer, ALB, and Hb between the two groups (*P* < 0.05), suggesting that they may have a merged influence on the development of gastrointestinal hemorrhage and cerebral infarction (Table 4).

### 3.6. Multivariate Logistic Regression Model to Analyze the Risk Factors of Cirrhosis Patients with Gastrointestinal Hemorrhage and Cerebral Infarction

Furthermore, a multivariate logistic regression model was used to analyze the risk factors of liver cirrhosis with gastrointestinal hemorrhage and cerebral infarction complications. The results showed significant differences in age, hypertension, bleeding history, infection, portal vein width, D-2 polymer, ALB, and Hb between the liver cirrhosis group and the combined gastrointestinal hemorrhage with cerebral infarction groups (*P* < 0.05, Table 5). The results indicate that they are all independent influencing factors of gastrointestinal hemorrhage combined with cerebral infarction complications in liver cirrhosis. Among them, age, hypertension, bleeding history, infection, portal vein width, and D-2 polymer were independent risk factors, and ALB and Hb hemoglobin were independent protective factors.

## 4. Discussion

Cirrhosis of the liver is a common digestive system disease with severe consequences in China. It is described as a chronic, progressive, and diffuse disease [17]. Upper gastrointestinal hemorrhage is one of the most common complications of liver cirrhosis [18] and presents as massive bleeding which easily leads to acute peripheral circulatory failure and a high mortality rate [19]. In the past, the mortality rate of liver cirrhosis complicated with upper gastrointestinal hemorrhage was 42.6%-65.0%. Among them, 40%-70% of patients died of the first hemorrhage, rebleeding occurred in 50%-80% of the patients treated with endoscopic hemostasis [20]. In this study, we found that the incidence of liver cirrhosis with gastrointestinal bleeding was 28.5%, which was consistent with the previous studies.

Liver cirrhosis patients are prone to thrombotic complications due to coagulation dysfunction, slow blood flow, and vascular endothelial damage [21]. Liver cirrhosis leads to an imbalance between coagulation factors and anticoagulation factors in the body; important anticoagulation factors such as antithrombin III (ATIII), protein C, and protein S are mainly synthesized by the liver. However, in patients with cirrhosis, the liver has decreased ability to synthesize such molecules, resulting in a hypercoagulable state. In patients with portal hypertension, the blood flow of the portal venous system is blocked, the blood flow velocity slows down, and even reverse blood flow occurs, which leads the portal venous system into a high-power, high-flow, and low-velocity stasis status with obstructed outflow tract. Vortex formation in the portal vein can cause vascular endothelial damage. All the above factors promote thrombosis [22, 23]. At the same time, patients with liver cirrhosis are prone to systemic infections due to poor nutritional status and reduced body function, such as abdominal cavity infections, respiratory tract, and skin infections resulting in obvious inflammatory reactions in the vascular intima. Such vascular conditions are conducive for thrombosis [24]. Cerebral embolism is usually caused by cardiogenic thrombosis [25]. The results of this study showed that 21.5% of patients with liver cirrhosis have a cerebral infarction. However, 11% of the patients with liver cirrhosis combined with gastrointestinal hemorrhage and cerebral infarction have the worst prognosis.

Owing to the associated risks of poor prognosis and mortality and a significant incidence of liver cirrhosis complications with gastrointestinal hemorrhage and venous thrombosis, it is necessary to determine the risk factors for their development in clinical practice. This will help in prediction and therefore early diagnosis and optimal treatment. Previous reports indicate that a history of bleeding from Esophageal Variceal Bleeding (EVB) is one of the causes of portal vein thrombosis in patients with liver cirrhosis [26]. In this study, in the single-factor analysis of patients with liver cirrhosis and cerebral infarction, we found that portal vein width, D-2 polymer, ALB, and Hb are predictors of liver cirrhosis with gastrointestinal hemorrhage and cerebral infarction. Age, alcohol consumption, bleeding history, and infection rates were observed to correlate with the occurrence of complications in patients with liver cirrhosis. In the further analysis of the unconditional logistic regression model of the risk factors of liver cirrhosis with gastrointestinal hemorrhage and cerebral infarction, it was found that the regression coefficients of the six variables of age, hypertension, bleeding history, infection, portal vein width, and D-2 polymers values were positive. The upper and lower limits of the 95% confidence interval were both >1, indicating that these 6 variables are all increased risk factors for patients with liver cirrhosis with gastrointestinal hemorrhage and cerebral infarction. These findings were consistent with those of previous studies where age, hypertension, infection, and a history of peptic ulcers were reported as risk factors for gastrointestinal hemorrhage and ischemic stroke in liver cirrhosis patients [27, 28]. In addition, age has been reported as a risk factor for gastrointestinal bleeding and ischemic stroke in the elderly [29, 30]. On the contrary, the ALB and Hb of the three complication groups were also significantly lower than those of the cirrhosis group and were determined as independent protection factors for mortality in liver cirrhosis with gastrointestinal hemorrhage and cerebral infarction complications.

## 5. Conclusion

In summary, age, hypertension, bleeding history, infection, portal vein width, and D-2 polymer are risk factors for gastrointestinal hemorrhage and cerebral infarction in patients with liver cirrhosis, while ALB and Hb are independent protective factors. This study provides a basis for improving the prognosis of patients with liver cirrhosis combined with gastrointestinal hemorrhage and cerebral infarction.

## Figures and Tables

**Figure 1:** Flowchart of the study.

**Figure 2:** Survival curve analysis of each group of patients.

**Figure 3:** The incidence of complications in patients with liver cirrhosis after 3, 6, 9, and 12 months of follow-up.

**Table 1:** General patient information.

Item	Liver cirrhosis group (*n* = 78)	Cerebral infarction group (*n* = 43)	Gastrointestinal hemorrhage group (*n* = 57)	Gastrointestinal hemorrhage with cerebral infarction group (*n* = 22)	*X* ^2^/*F*	*P*
Age (year)	48.51 ± 8.94	51.77 ± 11.68	54.12 ± 10.90^∗^	56.64 ± 10.37^∗^	5.226	0.002
Gender (%)					1.135	0.769
Male	56 (71.8)	33 (76.7)	39 (68.4)	17 (77.3)		
Female	22 (28.2)	10 (23.3)	18 (31.6)	5 (22.7)		
Height (cm)	165.19 ± 8.50	166.67 ± 9.33	167.91 ± 10.15	167.77 ± 8.31	1.124	0.340
Weight (kg)	64.27 ± 6.06	65.35 ± 6.11	65.61 ± 8.33	67.23 ± 6.05	1.218	0.304
BMI (kg/m^2^)	23.73 ± 3.22	23.69 ± 3.12	23.49 ± 3.79	23.98 ± 2.55	0.127	0.944
Duration of disease (year)	5.04 ± 4.93	5.16 ± 3.81	5.12 ± 5.18	5.43 ± 4.09	0.041	0.989
Heart rate (h)	66.91 ± 6.54	66.26 ± 7.76	66.46 ± 6.09	67.73 ± 6.93	0.281	0.839
Primary complications (%)					1.404	0.705
Without	66 (84.6)	35 (81.4)	44 (77.2)	17 (77.3)		
With	12 (15.4)	8 (18.6)	13 (22.8)	5 (22.7)		
Hypertension (%)					5.865	0.118
Without	67 (85.9)	31 (72.1)	41 (71.9)	15 (68.2)		
With	11 (14.1)	12 (27.9)	16 (28.1)	7 (31.8)		
Diabetes (%)					0.674	0.879
Without	66 (84.6)	35 (81.4)	47 (82.5)	17 (77.3)		
With	12 (15.4)	8 (18.6)	10 (17.5)	5 (22.7)		
Anemia (%)					0.208	0.976
Without	59 (75.6)	32 (74.4)	44 (77.2)	16 (72.7)		
With	19 (24.4)	11 (25.6)	13 (22.8)	6 (27.3)		
Arrhythmia (%)					3.391	0.335
Without	73 (93.6)	38 (88.4)	49 (86.0)	18 (81.8)		
With	5 (6.4)	5 (11.6)	8 (14.0)	4 (18.2)		
Alcohol consumption (%)					9.897	0.019
Without	68 (87.2)	30 (69.8)	43 (75.4)	13 (59.1)^∗^		
With	10 (12.8)	13 (30.2)	14 (24.6)	9 (40.9)^∗^		
Smoking (%)					5.223	0.156
Without	70 (89.7)	38 (88.4)	44 (77.2)	17 (77.3)		
With	8 (10.3)	5 (11.6)	13 (22.8)	5 (22.7)		
Ascites (%)					2.647	0.449
Without	62 (79.5)	29 (67.4)	45 (78.9)	16 (72.7)		
With	16 (20.5)	14 (32.6)	12 (21.1)	6 (27.3)		
History of bleeding (%)					10.277	0.016
Without	72 (92.3)	33 (76.7)^∗^	43 (75.4)^∗^	16 (72.7)^∗^		
With	6 (7.7)	10 (23.3)^∗^	14 (24.6)^∗^	6 (27.3)^∗^		
Hepatic encephalopathy (%)					2.323	0.508
Without	76 (97.4)	42 (97.7)	56 (98.2)	20 (90.9)		
With	2 (2.6)	1 (2.3)	1 (1.8)	2 (9.1)		
Infection (%)					18.779	0.001
Without	73 (93.6)	31 (72.1)^∗^	43 (75.4)^∗^	13 (59.1)^∗^		
With	5 (6.4)	12 (27.9)^∗^	14 (24.6)^∗^	9 (40.9)^∗^		
Surgical history (%)					1.695	0.638
Without	52 (66.7)	31 (72.1)	43 (75.4)	17 (77.3)		
With	26 (33.3)	12 (27.9)	14 (24.6)	5 (22.7)		
Arrhythmia (%)					1.192	0.755
Without	73 (93.6)	40 (93.0)	52 (91.2)	19 (86.4)		
With	5 (6.4)	3 (7.0)	5 (8.8)	3 (13.6)		

The data are expressed as mean ± SD or *n*(%). ^∗^*P* < 0.05 vs. liver cirrhosis group. BMI: body mass index.

**Table 2:** Comparison of clinical indicators among the four groups.

Item	Liver cirrhosis group (*n* = 78)	Cerebral infarction group (*n* = 43)	Gastrointestinal hemorrhage group (*n* = 57)	Gastrointestinal hemorrhage with cerebral infarction group (*n* = 22)	*F*	*P*
Portal vein width	1.26 ± 0.18	1.39 ± 0.20^∗^	1.35 ± 0.20^∗^	1.40 ± 0.20^∗^	6.334	0.001
Prothrombin time (PT)	13.41 ± 1.55	13.22 ± 1.59	13.37 ± 1.79	13.32 ± 1.93	0.124	0.946
D-2 polymer	0.40 ± 0.47	0.94 ± 1.14^∗^	0.48 ± 0.82^#^	1.09 ± 1.62^∗^^△^	5.621	0.001
Fibrinogen	2.49 ± 0.8	2.48 ± 0.79	2.51 ± 0.78	2.41 ± 0.58	0.096	0.962
Triglyceride (TG)	0.94 ± 0.45	1.00 ± 0.49	0.98 ± 0.45	1.02 ± 0.34	0.317	0.813
Total cholesterol (TC)	3.74 ± 1.19	3.44 ± 0.72	3.62 ± 1.03	3.93 ± 1.14	1.264	0.288
Low-density lipoprotein (LDL-C)	2.02 ± 0.77	1.81 ± 0.44	2.00 ± 0.68	2.08 ± 0.65	1.169	0.323
Alanine aminotransferase (ALT)	39.56 ± 25.14	34.91 ± 21.58	39.49 ± 29.47	41.91 ± 20.84	0.486	0.692
Aspartate aminotransferase (AST)	35.87 ± 25.02	33.84 ± 23.94	31.7 ± 14.65	34.14 ± 16.53	0.417	0.741
Albumin (ALB)	39.88 ± 4.86	35.97 ± 6.76^∗^	37.01 ± 5.04^∗^	33.6 ± 8.91^∗^^△^	8.514	0.001
Total bilirubin (TBIL)	20.84 ± 14.25	21.3 ± 14.91	18.17 ± 13.42	22.28 ± 11.45	0.710	0.547
Direct bilirubin (DBIL)	7.76 ± 6.54	7.61 ± 9.58	6.18 ± 5.48	7.53 ± 5.10	0.644	0.587
Blood urea nitrogen (BUN)	5.17 ± 1.89	4.89 ± 1.39	5.27 ± 1.47	5.30 ± 1.57	0.526	0.665
Creatinine (Cr)	72.54 ± 17.64	69.11 ± 11.73	73.11 ± 17.08	73.81 ± 16.05	0.661	0.577
C-reactive protein (CRP)	1.11 ± 1.21	1.41 ± 1.95	1.31 ± 1.52	1.62 ± 1.92	0.751	0.523
White blood cell count (WBC)	4.57 ± 1.54	4.34 ± 1.92	4.57 ± 1.73	4.60 ± 1.41	0.221	0.882
Platelet count (PLT)	111.99 ± 56.51	113.53 ± 68.61	119.54 ± 72.55	113.77 ± 51.05	0.164	0.921
Hemoglobin (Hb)	141.51 ± 23.26	130.49 ± 25.99^∗^	128.67 ± 22.74^∗^	127.23 ± 21.58^∗^	4.542	0.004

Data are expressed as mean ± SD. ^∗^*P* < 0.05 vs. cirrhosis alone group; ^#^*P* < 0.05 vs. cerebral infarction group; ^△^*P* < 0.05 vs. gastrointestinal hemorrhage group.

**Table 3:** Single-factor analysis to compare the basic situation between the two groups.

Item	Liver cirrhosis group (*n* = 78)	Gastrointestinal hemorrhage with cerebral infarction group (*n* = 122)	*X* ^2^/*t*	*P*
Age (year)	48.51 ± 8.94	53.75 ± 11.13	3.492	0.001
Gender (%)			0.032	0.858
Male	56 (71.8)	89 (73.0)		
Female	22 (28.2)	33 (27.0)		
Height (cm)	165.19 ± 8.50	167.45 ± 9.5	1.707	0.089
Weight (kg)	64.27 ± 6.06	65.81 ± 7.20	1.569	0.118
BMI (kg/m^2^)	23.73 ± 3.22	23.65 ± 3.35	0.163	0.871
Duration of disease (year)	5.04 ± 4.93	5.19 ± 4.51	0.224	0.823
Heart rate (h)	66.91 ± 6.54	66.61 ± 6.83	0.303	0.762
Primary complications (%)			1.086	0.297
Without	66 (84.6)	96 (78.7)		
With	12 (15.4)	26 (21.3)		
Hypertension (%)			5.716	0.017
Without	67 (85.9)	87 (71.3)		
With	11 (14.1)	35 (28.7)		
Diabetes (%)			0.396	0.529
Without	66 (84.6)	99 (81.1)		
With	12 (15.4)	23 (18.9)		
Anemia (%)			0.001	0.970
Without	59 (75.6)	92 (75.4)		
With	19 (24.4)	30 (24.6)		
Arrhythmia (%)			2.751	0.097
Without	73 (93.6)	105 (86.1)		
With	5 (6.4)	17 (13.9)		
Alcohol consumption (%)			7.482	0.006
Without	68 (87.2)	86 (70.5)		
With	10 (12.8)	36 (29.5)		
Smoking (%)			2.684	0.101
Without	70 (89.7)	99 (81.1)		
With	8 (10.3)	23 (18.9)		
Ascites (%)			0.852	0.356
Without	62 (79.5)	90 (73.8)		
With	16 (20.5)	32 (26.2)		
History of bleeding (%)			9.205	0.002
Without	72 (92.3)	92 (75.4)		
With	6 (7.7)	30 (24.6)		
Hepatic encephalopathy (%)			0.000	1.000
Without	76 (97.4)	118 (96.7)		
With	2 (2.6)	4 (3.3)		
Infection (%)			14.759	0.001
Without	73 (93.6)	87 (71.3)		
With	5 (6.4)	35 (28.7)		
Surgical history (%)			1.466	0.226
Without	52 (66.7)	91 (74.6)		
With	26 (33.3)	31 (25.4)		
Arrhythmia (%)			0.439	0.508
Without	73 (93.6)	111 (91.0)		
With	5 (6.4)	11 (9.0)		

The data are expressed as mean ± SD or *n*(%).

**Table 4:** Single-factor analysis compares clinical indicators between the two groups.

Item	Liver cirrhosis group (*n* = 78)	Gastrointestinal hemorrhage with cerebral infarction group (*n* = 122)	*t*	*P*
Portal vein width	1.26 ± 0.18	1.37 ± 0.20	4.167	0.001
Prothrombin time (PT)	13.41 ± 1.55	13.31 ± 1.74	0.434	0.665
D-2 polymer	0.40 ± 0.47	0.75 ± 1.14	2.630	0.009
Fibrinogen	2.49 ± 0.80	2.48 ± 0.75	0.039	0.969
Triglyceride (TG)	0.94 ± 0.45	0.99 ± 0.45	0.905	0.367
Total cholesterol (TC)	3.74 ± 1.19	3.62 ± 0.96	0.805	0.422
Low-density lipoprotein (LDL-C)	2.02 ± 0.77	1.95 ± 0.61	0.734	0.464
Alanine aminotransferase (ALT)	39.56 ± 25.14	38.31 ± 25.42	0.341	0.733
Aspartate aminotransferase (AST)	35.87 ± 25.02	32.89 ± 18.63	0.963	0.337
Albumin (ALB)	39.88 ± 4.86	36.03 ± 6.55	4.459	0.001
Total bilirubin (TBIL)	20.84 ± 14.25	20.01 ± 13.65	0.411	0.681
Direct bilirubin (DBIL)	7.76 ± 6.54	6.93 ± 7.12	0.830	0.408
Blood urea nitrogen (BUN)	5.17 ± 1.89	5.14 ± 1.46	0.125	0.900
Creatinine (Cr)	72.54 ± 17.64	71.83 ± 15.22	0.305	0.761
C-reactive protein (CRP)	1.11 ± 1.21	1.40 ± 1.75	1.273	0.204
White blood cell count (WBC)	4.57 ± 1.54	4.49 ± 1.74	0.320	0.750
Platelet count (PLT)	111.99 ± 56.51	116.39 ± 67.31	0.479	0.632
Hemoglobin (Hb)	141.51 ± 23.26	129.05 ± 23.58	3.665	0.001

**Table 5:** Multivariate logistic regression analysis.

Item	*B*	S.E.	Wald	*P*	OR	95% CI	
						Lower limit	Upper limit
Age	0.044	0.018	5.880	0.015	1.045	1.008	1.083
Hypertension	1.005	0.446	5.081	0.024	2.733	1.140	6.551
Alcohol consumption	0.414	0.488	0.717	0.397	1.512	0.581	3.939
Bleeding history	1.242	0.541	5.260	0.022	3.462	1.198	10.004
Infection	1.194	0.558	4.575	0.032	3.299	1.105	9.850
Portal vein width	2.154	1.008	4.568	0.033	8.616	1.196	62.084
D-2 polymer	0.543	0.256	4.492	0.034	1.720	1.042	2.841
ALB (albumin)	-0.082	0.037	4.993	0.025	0.921	0.858	0.990
Hb (hemoglobin)	-0.018	0.008	4.635	0.031	0.982	0.966	0.998

## Data Availability

The data used to support the findings of this study are available from the corresponding author upon request.

## Abbreviations

ALB: Albumin
ALT: Alanine aminotransferase
APTT: Activated partial prothrombin time
AST: Aspartate aminotransferase
BMI: Body mass index
B-ultrasound: Brightness-mode ultrasound
BUN: Blood urea nitrogen
Cr: Creatinine
CRP: C-reactive protein
CT: Computer tomography
DBIL: Direct bilirubin
Hb: Hemoglobin
LDL-C: Low-density lipoprotein
MRI: Magnetic resonance imaging
*N*: Number
PLT: Platelet count
PT: Prothrombin time
TBIL: Total bilirubin
TC: Total cholesterol
TG: Triglyceride
WBC: White blood cell count.
